This article has been retracted.

# Correlation of Serum IL-18, BDNF, and IL-1*β* with Depression and Prognosis after Acute Exacerbation of Chronic Obstructive Pulmonary Disease

**DOI:** 10.1155/2022/3555982

**Published:** 2022-04-30

**Authors:** Nan Zhao, Chengcheng Dong

**Affiliations:** Department of Respiration, The First Affiliated Hospital of Harbin Medical University, 150001 Harbin City, Heilongjiang Province, China

## Abstract

**Objective:**

To explore the correlation of serum IL-18, BDNF, and IL-1*β* with depression and prognosis after acute exacerbation of chronic obstructive pulmonary disease (COPD).

**Methods:**

By means of retrospective analysis, the data of 240 patients at the acute exacerbation of COPD treated in our hospital (February 2018-February 2021) were analyzed. All patients received conventional treatment 1 d after admission, patients' serological indicators were measured before treatment, and after 30 d of follow-up, the patients were divided into the survival group (SG) and death group (DG) according to their clinical outcomes, the Beck's Depression Inventory (BDI) scores of the surviving patients were investigated, the correlation of IL-18, BDNF, and IL-1*β* levels with depression was analyzed by R analytics, and the correlation of IL-18, BDNF, and IL-1*β* levels with prognosis was analyzed by ROC curve analysis.

**Results:**

The results of 30 d follow-up showed that 220 patients survived (91.7%) and 20 patients died (8.3%). Among the surviving patients, 95 patients had depression and 125 patients did not have depression; the BDI scores of the depressed subjects and the nondepressed subjects were 10.35 ± 1.25 points and 2.06 ± 0.76 points, respectively; significant differences in IL-18, BDNF, and IL-1*β* levels between SG and DG were observed (*P* < 0.05); significant differences in IL-18, BDNF, and IL-1*β* levels between the depressed subjects and the nondepressed subjects were observed (538.43 ± 19.02 vs. 515.32 ± 9.65, 7.54 ± 0.56 vs. 12.11 ± 2.41, and 8.70 ± 0.98 vs. 8.12 ± 0.87; *P* < 0.001); among the depressed patients, the IL-18 and IL-1*β* levels were positively correlative with the BDI scores (*r* = 0.781, *r* = 0.2583, *P* < 0.001, *P* = 0.012), and the BDNF level was negatively correlative with the BDI scores (*r* = −0.3277, *P* = 0.001) before treatment; according to the ROC analysis, the AUC (95% CI) of IL-18, BDNF, and IL-1*β* in predicting prognosis was 0.8770 (0.8281-0.9260), 0.7723 (0.6879-0.8567), and 0.7165 (0.6080-0.8250) (*P* < 0.05), respectively.

**Conclusion:**

In regard to the depression in COPD patients after acute exacerbation, IL18 and IL-1*β* show positive correlation, and BDNF presents negative correlation. All three indicators have predictive value for patient outcome.

## 1. Introduction

Chronic obstructive pulmonary disease (COPD) is a systemic disease characterized by persistent limitation of airflow, and its main pathological manifestation is chronic bronchitis; that is, various levels of bronchial wall are infiltrated by inflammatory cells, the accumulation of a large number of neutrophils can be seen after the disease enters the acute exacerbation stage, and in severe cases, it will evolve into suppurative inflammation, which causes the tracheal wall undergoing uninterrupted damage repair and then triggers tracheal remodeling [1–3]. The current worldwide incidence of COPD over the age of 40 has reached up to 10%, indicating that the disease has become a serious burden on the social medical field. Because early COPD is confined only to the lungs and can involve multiple organs with the development of inflammation, some scholars believe that COPD is the manifestation of a systemic inflammatory state in the lungs [4], and some argue that only “spillover” of inflammation will result in comorbidities [5]. Inflammatory factors are messengers linking the immune system to the central system, so most comorbidities of COPD, such as depression, are characterized by high levels of inflammatory factors [6]. Depression is one of the most frequent comorbidities in COPD patients, but its incidence varies widely in different studies. Foruhar et al. found that the probability of concurrent depression in COPD patients can reach 79.0% [7] and speculated that its incidence is correlated with patients' levels of inflammatory factors. The relationship between depression and inflammatory factors has been confirmed by domestic and foreign published works [8], and immune factors, mainly divided into proinflammatory cytokines and anti-inflammatory cytokines, are important in the occurrence and development of depression, but whether the levels of inflammatory factors in COPD patients can affect the incidence of depression remains inconclusive in academia. Scholars Zhang et al. found that patients with higher levels of tumor necrosis factor *α* (TNF-*α*) and interleukin-6 (IL-6) are prone to depression and that TNF-*α* and IL-6 show a positive association with the occurrence of depression [9]; i.e., the lower the level of inflammatory factors, the less likely the patient has concurrent depression. However, the key inflammatory indicators of COPD are not limited to TNF-*α* and IL-6, and theoretical research on the correlation between the levels of inflammatory factors and the onset of depression after acute exacerbation in COPD patients remains blank. IL-18 and IL-1*β* were selected as the inflammation indicators in this study; both are strongly linked to the onset and progress of COPD, in which IL-18 is an important class of proinflammatory factors that can induce macrophage and lymphocyte infiltration and accelerate vascular remodeling, while IL-1*β* can activate the MAPK signaling pathway, thereby increasing the expression of a series of inflammation-related factors [10] and aggravating the condition of patients. On this basis, BDNF was selected as a relevant factor for depression, which is a protein with pronerve growth activity that can maintain the activation of detoxification/antioxidant enzymes in a highly expressed manner, thus maintaining a preventive mechanism against depression [11]. The study was aimed at further exploring the correlation of levels of inflammatory factors with depression and prognosis by analyzing the outcomes of 240 COPD patients after 30 d, so as to provide more clinical reference basis.

## 2. Materials and Methods

### 2.1. Study Design

This retrospective study was conducted under the guidance of the *World Medical Association Declaration of Helsinki (2013)* [12] to explore the correlation of serum IL-18, BDNF, and IL-1*β* with depression and prognosis after acute exacerbation of COPD.

### 2.2. General Data

Inclusion criteria are as follows: (1) the patients were diagnosed with COPD after physical examination, lung function examination, and imaging examination, met the diagnosis criteria in the *Guidelines for the Diagnosis of Chronic Obstructive Pulmonary Disease* [13], and were admitted to the hospital within 48 h of exacerbation; (2) the patients accepted standardized therapy after admission and were discharged after their condition was stable; (3) the patients accepted 30 d of follow-up after discharge; (4) the patients did not have history of depression before suffering from COPD; (5) the patients did not receive antidepression treatment before admission; (6) the patients were over 18 years old; and (7) the patients had complete clinical data.

Exclusion criteria are as follows: (1) the patients were complicated with other diseases that may affect the study results; (2) the patients quit the treatment in the middle of the study; (3) the patients had a family history of mental illness; (4) the patients suffered from depression caused by organic mental disorders or psychoactive substance; (5) the patients received surgery within 15 d before admission; and (6) the patients were pregnant or lactating women.

According to the above criteria, 240 COPD patients treated in our hospital (February 2018-February 2021) were selected, including 130 males and 110 females, with a mean age of 60.42 ± 5.41 years, and there were 90 mild cases, 110 moderate cases, and 40 severe cases. All patients understood the study objective and signed the informed consent.

### 2.3. Methods

#### 2.3.1. Treatments

After admission, patients in the two groups received oxygen inhalation, anti-inflammation, relieving cough and asthma, and fluid infusion treatments, and at the same time, their water and electrolyte balance was maintained. The patients daily inhaled 2.5 mL of salbutamol sulfate solution (manufacturer: Yangzhou No. 3 Pharmaceutical Co., Ltd.; NMPA approval no. H20123384), 2.0 mL of budesonide suspension liquid (manufacturer: Sichuan Purity Pharmaceutical Co., Ltd.; NMPA approval no. H20213286), and 2.0 mL of ipratropium bromide solution (manufacturer: Sichuan Purity Pharmaceutical Co., Ltd.; NMPA approval no. H20203591), twice a day for 7-14 d, and were discharged after their condition was stable. After discharge, patients continued to receive conventional drug treatment by daily inhaling 18 *μ*g of tiotropium bromide powder for inhalation (manufacturer: Chia Tai Tianqing Pharmaceutical Group Co., Ltd.; NMPA approval no. H20060454) once and orally taking 0.5 g of corbrin capsule (manufacturer: Hangzhou Zhongmei Huadong Pharmaceutical Co., Ltd.; NMPA approval no. Z10910036) three times.

#### 2.3.2. Serological Test

Before treatment, 3 mL of fasting elbow venous blood was drawn from the patients in the morning to centrifuge 15 min under 3,500 r/min and take the supernatant for test. After collecting all specimen, the levels of serum IL-18, BDNF, and IL-1*β* were measured by enzyme-linked immunosorbent assay (Beijing Kewei Clinical Diagnostic Reagent Inc.; NMPA approval no. S20060028).

#### 2.3.3. Investigation Methods

After discharge, 30 d follow-up was conducted, and the patients were divided into the survival group (SG) and death group (DG) according to their clinical outcomes. The patients in SG were scored with the Beck's Depression Inventory (BDI) [14], which contained 13 items related to depression, each item was rated on a scale of 0-3 points, and the total score of the inventory was 39 points, with ≥5 points indicating depression. The surviving patients were subdivided into the depressed subjects and nondepressed subjects; the levels of inflammatory factors were compared between SG and DG as well as between depressed and nondepressed subjects, so as to analyze the relationship between the levels of inflammatory factors and depression and prognosis of patients.

### 2.4. Statistical Processing

In this study, the data processing software was SPSS20.0, the picture drawing software was GraphPad Prism 7 (GraphPad Software, San Diego, USA), the items included were enumeration data and measurement data, the correlation of IL-18, BDNF, and IL-1*β* levels with depression was analyzed by R analytics, the correlation of IL-18, BDNF, and IL-1*β* levels with prognosis was analyzed with the ROC curves, and differences were considered statistically significant at *P* < 0.05.

## 3. Results

### 3.1. Patient Grouping

The results of 30 d follow-up showed that 220 patients survived and 20 patients died. Among the surviving patients, there were 115 males and 105 females, 95 patients had depression, and 125 patients did not have depression. The depression group had 50 males and 45 females, and the BDI score was 10.35 ± 1.25 points; and the nondepression group had 65 males and 60 females, and the BDI scores of was 2.06 ± 0.76 points.

### 3.2. Comparison of Patients' IL-18, BDNF, and IL-1*β* Levels

Figure 1 showed that the IL-18, BDNF, and IL-1*β* levels were significantly different between SG and DG (*P* < 0.05) as well as between depressed and nondepressed subjects (*P* < 0.001).

Before treatment, the IL-18, BDNF, and IL-1*β* levels were significantly different between SG and DG (525.30 ± 18.44 vs. 550.32 ± 9.64, 10.14 ± 2.92 vs. 13.11 ± 2.41, and 8.37 ± 0.97 vs. 9.00 ± 0.80; *P* < 0.05); and the IL-18, BDNF, and IL-1*β* levels were significantly different between depressed and nondepressed subjects (538.43 ± 19.02 vs. 515.32 ± 9.65, 7.54 ± 0.56 vs. 12.11 ± 2.41, and 8.70 ± 0.98 vs. 8.12 ± 0.87; *P* < 0.001).

### 3.3. Correlation of IL-18, BDNF, and IL-1*β* Levels with Depression and Prognosis

The correlation analysis showed that before treatment, the IL-18 and IL-1*β* levels were positively correlative with the BDI scores (*r* = 0.781, *r* = 0.2583, *P* < 0.001, *P* = 0.012), and the BDNF level was negatively correlative with the BDI scores (*r* = −0.3277, *P* = 0.001) in the depression group (see Figure 2).

The ROC analysis showed that the AUC (95% CI) of IL-18, BDNF, and IL-1*β* in predicting prognosis was 0.8770 (0.8281-0.9260), 0.7723 (0.6879-0.8567), and 0.7165 (0.6080-0.8250) (*P* < 0.05), respectively (see Figure 3).

## 4. Discussion

Depression is a common psychopathological syndrome, and its occurrence is closely related to social, psychological, and biological factors [15]. In a study involving 18,588 COPD patients, scholars Schane et al. found that approximately 40.0% of patients had symptoms of depression, which was significantly higher than the probability of stroke, diabetes mellitus, arthritis, and other chronic diseases [16], and that depression would increase the likelihood of readmission and death in COPD patients, affecting patient outcomes. The data in 2019 show that the prevalence of depression reached 2.1% in China, indicating that depression has become an important psychological and psychiatric disease affecting residents' quality of life. However, there are fewer patients with COPD complicated by depression, so no attention has been paid to the clinical diagnosis of COPD patients with depression, thus making the treatment of patients delayed. With the continuous development of psychoimmunology at the current stage, more and more studies have shown that cytokines may be critical to in the occurrence and development of depression [17, 18], and the reason why COPD patients have concurrent depression is similarly closely related to cytokines. Immune factors are cellular molecules secreted by immunocompetent cells that have a bioactive role in regulating immune responses and are mainly divided into proinflammatory cytokines and anti-inflammatory cytokines. After the immune response system is activated, the human body will release proinflammatory cytokines, causing neuroendocrine and neurobiological changes, and IL-1, IL-6, and other factors can reduce neuroplasticity by directly stimulating the hypothalamic-pituitary-adrenal axis and accelerate tryptophan breakdown, the precursor substance of 5-hydroxytryptamine, thus participating in the pathogenesis of depression [19, 20]. Depending on the molecular structure, IL-1 can be subdivided into IL-1*α* and IL-1*β*, of which IL-1*β* is closely related to autoinflammatory and autoimmune diseases and can act with the coreceptor IL-1RacP to form a complex, activate the MAPK signaling pathway within target cells, and induce inflammatory factors expression [21]. Reports have shown that IL-1*β* in COPD patients presented in an aggregated state, whereas blockade of IL-1*β* could alleviate the clinical symptoms of patients [22], indicating that IL-1*β* can affect patient outcomes. In this study, the 30 d follow-up results showed 220 surviving patients and 20 dead patients, and patients with different outcomes had obviously varied IL-1*β* levels, with AUC (95%CI) = 0.7165 (0.6080-0.8250) for this indicator to predict prognosis, confirming that IL-1*β* is associated with patient outcomes. Not only that, some scholars found that IL-1*β* level increased in peripheral blood of depression model rats and the depressive manifestations of rats improved after antagonist injection [23]. This study concluded that IL-1*β* was positively correlated with BDI score (*r* = 0.2583, *P* = 0.012), and therefore, IL-1*β* is an inflammatory factor with an important role in COPD complicated with depression.

In addition to IL-1*β*, IL-18 is also significant in the onset and progress of COPD. IL-18, a pro-inflammatory factor, is able to promote T lymphocyte proliferation while inducing an immune response dominated by Th1 cells, and this indicator showed a positive correlation with the expression of NLRP3 mRNA [24]. The NLRP3 inflammasome is a component of the human immune system, factors such as smoke exposure and infection can trigger systemic inflammatory responses via the NLRP3 signaling pathway, and overactivated NLRP3 signaling can upregulate IL-18 content and thus accelerate COPD development, so IL-18 levels can reflect the severity of patients' conditions. In this study, it was found that the IL-18 level in SG was significantly different from that in DG (*P* < 0.05), and the IL-18 level in depressed subjects was significantly different from that in nondepressed subjects (*P* < 0.001), indicating that this indicator is strongly related to patients' depression and prognosis. This argument was further confirmed by the ROC curve and R analytics, with AUC (95%CI) = 0.8770 (0.8281-0.9260) for IL-18 to predict prognosis and a positive correlation between pretreatment IL-18 levels and BDI scores in depressed subjects (*r* = 0.781, *P* < 0.001); that is, the higher the IL-18 level, the more likely the patients are to have concurrent depression. In this study, 95 patients had depression, with a probability of 43.2%, the BDNF level of depressed patients was lower than that of nondepressed patients, and this indicator showed a negative correlation with BDI scores (*r* = −0.3277, *P* = 0.001), owing to the fact that BDNF can control the nuclear translocation of the redox-sensitive transcription nuclear factor erythroid 2-related factor 2 (Nrf2), a master regulator of redox homeostasis. High BDNF levels can accelerate Nrf2 translocation, which elevates the activity of antioxidant enzymes and inhibits oxidative stress, making patients less susceptible to depression. The correlation between BDNF and depression has been confirmed by literature [25]. BDNF is expressed in brain tissue, and its levels will be further elevated when platelets are affected by thrombin. BDNF levels are reduced in depressed patients and negatively correlate with the severity of the condition. ROC analysis showed that the AUC (95%CI) = 0.7723 (0.6879-0.8567) of BDNF in predicting prognosis of COPD patients, indicating the value of BDNF in this regard, but the mechanism is not clear and may be related to depression of patients, so further exploration and research are needed.

## 5. Conclusion

To sum up, in regard to the depression in COPD patients after acute exacerbation, IL18 and IL-1*β* show positive correlation, and BDNF presents negative correlation. All three indicators have predictive value for patient outcome. Clinically, patient prognosis can be predicted by IL-18, IL-1*β* and BDNF, so as to perform corresponding intervention measures.

## Figures and Tables

**Figure 1:** Comparison of patients' IL-18, BDNF, and IL-1*β* levels (±s). Note: (a) denoted IL-18 (pg/mL); (b) denoted BDNF (*μ*g/L); and (c) denoted IL-1*β* (pg/mL).

**Figure 2:** Correlation of IL-18, BDNF, and IL-1*β* levels with depression.

**Figure 3:** Correlation of IL-18, BDNF, and IL-1*β* levels with prognosis.

## Data Availability

The data to support the findings of this study is available on reasonable request from the corresponding author.
